RETRACTED

# Propofol modulates glycolysis reprogramming of ovarian tumor via restraining circular RNA-zinc finger RNA-binding protein/microRNA-212-5p/superoxide dismutase 2 axis

**DOI:** 10.1080/21655979.2022.2063649

**Published:** 2022-05-11

**Authors:** DongDong Qu, Xin Zou, ZhiLin Liu

**Affiliations:** a Department of Anesthesiology, Jinan Maternal and Child Health Hospital, Jinan City, Shandong Province, China; b Department of Anesthesiology, Qingdao Women’s and Children’s Hospital, Qingdao City, Shandong Province, China; c Department of Anesthesiology, Qingdao Municipal Hospital Affiliated to Qingdao University, Qingdao City, Shandong Province, China

**Keywords:** Ovarian tumor, Propofol, circular-ZFRS, MicroRNA-212-5p, superoxide dismutase 2, glycolysis reprogramming

## Abstract

Metabolic reprogramming refers to the transformation of the whole metabolic network covering glycolysis and mitochondrial metabolism, which is primarily manifested as the Warburg effect and mitochondrial metabolic reprogramming. Propofol (Pro) has been testified to suppress the malignancy of diversified human cancers. Nevertheless, its role in glycolysis is still uncertain. The purpose of this study was to determine whether Pro modulated glycolysis in ovarian cancer (OC) cells. Cell proliferation, apoptosis, migration, and invasion were tested via CCK-8, flow cytometry, and Transwell assays, respectively, and glucose intake, lactic acid, and ATP production were also determined. Pro restrained glycolysis via mediating the circular RNA-zinc finger RNA-binding protein (ZFR)/microRNA (miR)-212-5p/superoxide dismutase 2 (SOD2) axis. Additionally, Pro restrained cancer cell advancement via modulating circ-ZFR/miR-212-5p/SOD2 axis. In short, Pro restrained glycolysis via mediating the circ-ZFR/miR-212-5p/SOD2 axis. These results offered a better theoretical foundation for comprehending the molecular pathology of OC and provided a novel target for OC diagnosis and treatment.

## Highlights

- Pro inhibits OC cell growth and glycolysis;
- Pro reduces circ-ZFR expression to elevate miR-212-5p expression;
- circ-ZFR silencing or miR-212-5p overexpression inhibits OC cell growth and glycolysis;
- miR-212-5p targets SOD2.
- Pro by regulating circ-ZFR/miR-212-5p/SOD2 axis inhibits OC development.

## 1 Introduction

Ovarian cancer (OC) is an extremely invasive and metastatic gynecological malignant tumor with a 5-year survival rate of approximately 47% and a local staging diagnosis rate of 15% [1]. Numerous patients are only diagnosed until the disease reaches an advanced stage owing to the lack of available biomarkers to precisely detect the illness [2]. At present, the critical clinical treatment methods for OC cover surgery, immunotherapy, and chemotherapy. These strategies prolong patients’ survival time to some extent, but OC prognosis is still unpleasing and the risk of recurrence is high [3]. It is urgent to explore OC’s pathogenesis, which is critical to developing novel biomarkers and curative drugs for OC diagnosis and prognosis.

RETRACTED

Numerous evidence has clarified anesthetics are available to enhance long-term survival and prevent cancer recurrence after surgery [4]. Propofol (Pro) is a hypnotic alkyl phenol derivative with diversified biological activities and is an extremely prevalent intravenous anesthetic in clinical practice [4]. Researchers have elucidated Pro is provided with anticancer activity, which is available to restrain cancer cell advancement and sensitize cancer cells to chemotherapy, and is provided with anti-tumor effects in diversified cancers, covering colorectal cancer (CRC) [5], pancreatic cancer [6], gastric cancer (GC) [7] and OC [8]. Nevertheless, the latent mechanism of Pro in cancer remains unknown. Otto Heinrich Warburg discovered the aberrant metabolic behavior of tumor cells in 1920, that is, cancer cells are more prone to gain energy via aerobic glycolysis (AG) vs. oxidative phosphorylation even under aerobic conditions, which is also known as the Warburg effect [9]. AG is conducive to the rapid generation of energy, biosynthesis, and treatment resistance and accelerates the sustaining cancer cell advancement, thereby boosting cancer’s malignant development [10]. Consequently, targeting glucose metabolism reprogramming is available to be the latent approach for OC therapy [11].

There is a large number of non-encoded RNA (ncRNAs) involved in the progression of propofol-mediated cancer [PMID:29628875] [PMID: 31,297,532]. Circular RNAs (circRNAs), a class of conserved non-coding RNA with a closed-loop structure, broadly exist in diversified eukaryotes, and are generated via multiple protein-coding genes in superior eukaryotes via reverse splicing of exons [12]. CircRNA’s dysregulation is associated with multiple illnesses’ occurrence and advancement, covering cancer. Additionally, circRNAs generally exert critical biological functions via performing as microRNA sponges to modulate target mRNA [13]. Circ-zinc finger RNA-binding protein (ZFR), a newly identified circRNA, has been testified to be elevated in bladder cancer (BC) [14] and boost BC cell advancement via augmenting WNT5A signal to absorb miR-545 and miR-1270. Nevertheless, circ-ZFR’s action in OC remains unknown.

MicroRNAs (miRNAs) are small non-encoded RNAs that transcriptionally regulate the expression of mRNAs. MiRNAs could act on cell cycle, apoptosis, and differentiation [PMID: 28,209,991] and function as carcinogenic miRNAs and tumor inhibition miRNAs [PMID: 27,795,564]. miR-212 on chromosome 17P13.3 is disordered in several human cancers [PMID: 28,504,814] and could suppress tumor growth in non-small cell lung cancer [PMID: 23,974,008]. However, other studies have shown that miR-212 exhibits carcinogenic properties in colorectal cancer and pancreatic cancer [PMID: 26,692,142] [PMID: 27,814,273]. Therefore, the biological function of miR-212 is cancer-specific, partly because of the different cellular environments of various tumors. Nevertheless, the role of miR-212-5p in OC has not been determined.

RETRACTED

In this research, the latent role of Pro in OC’s AG and the association of Pro with circ-ZFR were primarily explored. In *vitro* cell experiments testified Pro-restrained OC progression via suppressing AG and uncovered the molecular mechanism of Pro with the involvement of circ-ZFR/miR-212-5p/superoxide dismutase 2 (SOD2) axis.

## 2 Materials and methods

### 2.1 Cell culture

The purchase of human OC cell line A2780 was by the American Type Culture Collection Center. A2780 cells were replenished with Dulbecco’s Modified Eagle Medium (DMEM) with 10% Fetal bovine serum (FBS) (Gibco; Thermo Fisher Scientific, Inc.) and maintained in the humid atmosphere until 80–90% confluence.

### 2.2 Pro treatment

Pro was purchased from Sigma-Aldrich (Merck KGaA), dissolved in dimethyl sulfoxide (Sigma-Aldrich), and stored at −20°C. OC cells were treated with 0, 5, 10, or 20 μg/mL Pro.

### 2.3 Cell transfection

Synthesis of short hairpin small interfering RNA (sh-ZFR: 5’-TCAAATTTATGCCCAGCCGGC-3’) and its negative control (NC) (sh-NC: 5’-TTCTCCGAACGTGTCACGT-3’) of targeting circ-ZFR and miR-212-5p mimic (5’-ACCUUGGCUCUAGACUGCUUACU-3’) and its NC (mimic NC) (5’-UUCUCCGAACGUGUCACGUTT-3’) was performed (Shanghai Gene Pharmaceutical Co., Ltd.). The full-length SOD2 sequence was amplified and connected to the pcDNA3.1 plasmid (OriGene Technologies, Inc.), and the plasmid after recombining was named PCDNA3.1-SOD2. Transfection of the cells was by Lipofectamine 2000 reagent (Invitrogen; Thermo Fisher Scientific, Inc.) in light of the manufacturers’ protocol. Subsequently, the cells were treated with 20 μg/mL Pro.

### 2.4 Cell counting kit-8 (CCK-8)

In brief, 1 × 10^4^ cells were seeded into 96-well plates, and 10 μL CCK-8 solution (Beyotime Institute of Biotechnology) was added to each well after Pro treatment or transfection. After incubation, measurement of absorbance was performed at 490 nm on a spectrophotometer.

### 2.5 Flow cytometry

For cell apoptosis analysis, seeding of cells with different treatments was in 6-well plates with 3 × 10^5^ cells per well without FBS. The cells were then gained and stained with fluorescein isothiocyanate-coupled annexin V and propidium iodide (BD Pharmingen) in line with the manufacturer’s instructions. Determination of apoptotic cells was by FACS Flow Cytometry (BD Biosciences, Franklin Lakes, NJ, USA).

RETRACTED

### 2.6 Transwell

Cell invasion experiment was implemented in a Transwell cell culture chamber (Millipore, Billerica, MA, USA) coated with Matrigel. Cells (1 × 10^5^) were placed into the upper chamber coated with 150 mg Matrigel (BD Biosciences, Bedford, MD, USA). The lower chamber was filled with DMEM covering 10% FBS. After incubation, removal of residual cells on the upper surface of the membrane was conducted. The cells fixed on the lower surface of the membrane were stained with crystal violet. Photos were taken under a microscope (Olympus). In the cell migration experiment, no Matrigel coating was needed on the upper chamber of the Transwell chamber, and the other operations were the same as the invasion experiment.

### 2.7 Glucose uptake, lactic acid and adenosine triphosphate (ATP) determination

Examination of glucose uptake, lactic acid, and ATP production in HeLa cells was conducted via glucose uptake colorimetric assay kit (Biovision, Milpitas, CA, USA), lactic acid assay kit (Sigma St. Louis, MO, USA), and ATP colorimetric kit (Sigma).

### 2.8 Reverse transcription quantitative polymerase chain reaction (RT-qPCR)

Extraction of total RNA was from tissues and cell lines adopting TRIzol reagent (Thermo Fisher Scientific, Inc.) in light of the manufacturer’s instructions. A total of 1 μg RNA was transformed into a complementary DNA adopting the SuperScript one-step RT-PCR kit (Thermo Fisher Scientific, Inc.) in light of the manufacturer’s instructions. RT-qPCR was implemented in ABI 7500 FLUORESCENCE qPCR machine (Applied Biosystems; Thermo Fisher Scientific, Inc.) adopting the Applied Biosystems™ PowerUp™ SYBR Green Master Mix kit (Thermo Fisher Scientific, Inc.). U6 and glyceraldehyde-3-phosphate dehydrogenase (GAPDH) were loading controls. Calculation of each gene’s relative quantitative values was by 2^−ΔΔCt^ method. Primer sequences (GenePharma Co., Ltd., Shanghai, China) are presented in Table 1.

**Table 1.** Primers for RT-qPCR

Genes	Primer sequences (5’–3’)
Circ-ZFR	F: TCCCAATGCTAAGGAGATGC
	R: TTCTTCTCGTCTTCGCCAGT
MiR-212-5p	F: ACCTTGGCTCTAGACTGCT
	R: GCAGGGTCCGAGGTATTC
SOD2	F: GCCTCCCTGACCTGCCTTAC
	R: GTGATTGATATGGCCCCCG
U6	F: CTCGCTTCGGCAGCACA
	R: AACGCTTCACGAATTTGCGT
GAPDH	F: CGGAGTCAACGGATTTGGTCGTAT
	R: AGCCTTCTCCATGGTGGTGAAGAC

### 2.9 Western blot

Extraction of proteins was by a Radio-Immunoprecipitation assay lysis buffer (Beyotime, Haimen, China). Qualification of the protein concentration was via bicinchoninic acid (BCA) protein determination kit (Beyotime). The same amount of protein was separated via sulfate polyacrylamide gel electrophoresis, electroblotted onto polyvinylidene fluoride membrane (Bio-Rad, Hercules, CA, USA) and blocked. The membranes were incubated with primary antibodies SOD2 (AB13533, 1:1000, Abcam), cleaved-PARP (1:1000, Cell Signaling Technology) and GAPDH (AB8245, 1:1000, Abcam), and with horseradish peroxidase coupled secondary antibody. Testing of blot was conducted via the electrogenerated chemiluminescence detection system.

RETRACTED

### 2.10 The luciferase activity assay

The binding sites of miR-212-5p with circ-ZFR or SOD2 were predicted via starBase. The wild type (WT) and mutant (MUT) fragments of circ-ZFR were cloned into pGLO vector (GenScript, Nanjing, China) to construct circ-ZFR-WT and circ-ZFR-MUT plasmids. The 3’-untranslated region sequence of SOD2 covering a predicted or mutated miR-212-5p binding site was used to construct SOD2-WT/MUT plasmids. The cells were co-transfected with miR-212-5p mimic (12.5 or 25 pmol per well) or mimic NC (12.5 or 25 pmol per well) and the corresponding reporter plasmid (0.5 μg per well) adopting Lipofectamine^TM^ 2000 (Invitrogen). After a transfection of 48 h, examination of luciferase activity was dependent on luciferase detection kit (KeyGEN, Jiangsu, China).

### RNA immunoprecipitation (RIP)

RIP assay was conducted as previously described [PMID:28887321]. A2780 cells (2 × 10^7^) were collected to perform RIP assay using 5  μg AGO2 antibody (Millipore, MA, USA) or normal rabbit IgG. The co-precipitated RNAs were isolated and detected by RT-qPCR.

### 2.11 Statistical analysis

Statistical analysis was implemented via SPSS 19.0 software (IBM Corp.). Graphs were drawn via GraphPad Prism 6 Software (GraphPad Software, Inc.). Comparison of two or more groups was conducted via a two-tailed paired Student’s t test and a one-way analysis of variance (ANOVA), respectively. Verification of pairwise comparisons of ANOVA was by Tukey’s postmortem test. *P* < 0.05 was accepted as indicative of distinct differences.

## 3 Results

### 3.1 Pro restrains OC cell advancement with glycolysis

To investigate the effect of Pro on A2780 cells, A2780 cells were treated with 0, 5, 10, and 20 μg/mL Pro, and the cell viability and apoptosis rate were determined. The results showed that Pro had a significant dose-dependent inhibitory effect on cell viability and a significant dose-dependent promotion effect on the apoptosis rate of A2780 cells (Figure 1(a, b)). By immunoblotting for the apoptosis marker CLEAVED-PARP, it was determined that Pro significantly promoted Cleaved-PARP expression in a dose-dependent manner (Figure 1(c)). Cell migration and invasion were detected by Transwell, and Pro was found to inhibit the migration and invasion of A2780 cells in a dose-dependent manner (Figure 1(d, e)). Measurements of glycolysis indicated that glucose intake, lactic acid, and ATP were reduced as the Pro concentration increased (figure 1(f)). To determine the association of Pro dose with circ-ZFR, CiRC-ZFR expression under different concentrations of Pro was checked by RT-qPCR, and results showed that Pro significantly reduced CiRC-ZFR expression in A2780 cells in a dose-dependent manner (Figure 1(g)). Consequently, 20 μg/mL Pro was used for subsequent experiments.

RETRACTED

**Figure 1.** Pro constrains OC cell advancement with glycolysis.

a. CCK-8 detection of cell proliferation; b. Flow cytometry test of cell apoptosis; c. Western blot analysis of cleaved-PARP expression; d-e. Transwell examination of cell migration and invasion; f. Glucose uptake, lactic acid, and ATP production; g. RT-qPCR test of circ-ZFR. The data in the figure were all measurement data, and the manifestation of the values was in mean ± standard deviation (SD) (N = 3). * Vs. the 0 μg/mL, *P* < 0.05.

### 3.2 Repressive circ-ZFR constraints OC cell advancement with glycolysis

RT-qPCR results proved that circ-ZFR expression could be lowered by Pro. To further determine circ-ZFR’s influence on A2780 cells, transfection of sh-ZFR, and its NC (sh-NC) was performed in A2780 cells treated with 20 μg/mL Pro. The sh-ZFR distinctly declined circ-ZFR expression (Figure 2(a)). A2780 cell advancement with glycolysis was repressed after silencing circ-ZFR (Figure 2(b-g)). To sum up, suppressing circ-ZFR expression constrained OC cell progression with glycolysis.

**Figure 2.** Repressive circ-ZFR constraints OC cell progression with glycolysis.

a. RT-qPCR test of circ-ZFR; b. CCK-8 detection of cell proliferation; c. Flow cytometry examination of cell apoptosis; d. Western blot analysis of cleaved-PARP expression; e-f. Transwell test of cell migration and invasion; g. Glucose uptake, lactic acid, and ATP production. The data in the figure were all measurement data, and the manifestation of the values was in mean ± SD (N = 3). * Vs. the Control; *P* < 0.05; # Vs. the Pro + sh-NC;*P* < 0.05.

### 3.3 Circ-ZFR negatively modulates miR-212-5p

To further determine the regulatory mechanism of circ-ZFR, the downstream targets of circ-ZFR were explored in this research. StarBase predicted the binding site of circ-ZFR and miR-212-5p (Figure 3(a)). Luciferase activity was critically reduced in cells after co-transfection with circ-ZFR-WT and miR-212-5p mimic (Figure 3(b)). RIP experiments exhibited that circ-ZFR and miR-212-5p can be rich in Anti-AGO2 (Figure 3(c)). Additionally, silenced circ-ZFR distinctively elevated miR-212-5p expression in A2780 cells (Figure 3(d)). Consequently, circ-ZFR might combine with miR-212-5p and negatively modulate its expression.

RETRACTED

**Figure 3.** Circ-ZFR negatively modulates miR-212-5p.

a. StarBase forecast of the binding site of circ-ZFR with miR-212-5p; b. The luciferase activity verification of the binding of circ-ZFR with miR-212-5p; c. RIP detection of the relation between Circ-ZFR and miR-212-5p; D. RT-qPCR detection of miR-212-5p. The data in the figure were all measurement data, and the manifestation of the values was mean ± SD (N = 3). * Vs. the Control; *P* < 0.05; # Vs the Pro + sh-NC;*P* < 0.05.

### 3.4 Elevated miR-212-5p represses OC cell advancement with glycolysis

To further determine miR-212-5p’s influence on A2780 cells, transfection of miR-212-5p mimic and its NC (mimic NC) was carried out in A2780 cells treated with 20 μg/mL Pro, and verification of the transfection efficacy was implemented (Figure 4(a)). The experimental results elucidated that A2780 cells progression and glycolysis were constrained after elevating miR-212-5p expression (Figure 4(b-g)). In brief, augmenting miR-212-5p expression suppressed OC cell advancement with glycolysis.

**Figure 4.** Elevated miR-212-5p restrains OC cell progression with glycolysis.

a. RT-qPCR test of miR-212-5p; b. CCK-8 detection of cell proliferation; c. Flow cytometry examination of cell apoptosis; d. Western blot analysis of cleaved-PARP expression; e-f. Transwell detection of cell migration and invasion; g. Glucose uptake, lactic acid, and ATP production. The data in the figure were all measurement data, and the manifestation of the values was mean ± SD (N = 3). * Vs the Pro + mimic NC, *P* < 0.05.

### 3.5 MiR-212-5p targets SOD2

To further determine the regulatory mechanism of miR-212-5p, the downstream target genes of miR-212-5p were explored in this research, and verification of the association between miRNA and target genes was implemented. StarBase predicted the targeting site of miR-212-5p and SOD2 (Figure 5(a)). Luciferase activity was critically declined in cells after co-transfection with SOD2-WT and MiR-212-5p mimic (Figure 5(b)). RIP assay demonstrated that miR-212-5p and SOD2 mRNA could be enriched by anti-Ago2 (Figure 5(c)). Additionally, elevated miR-212-5p distinctively constrained SOD2 expression in A2780 cells (Figure 5(d)). To sum up, miR-212-5p targeted SOD2.

**Figure 5.** MiR-212-5p targets SOD2.

a. StarBase forecast of the target sites of miR-212-5p with SOD2; b. The luciferase activity verification of the targeting of miR-212-5p with SOD2; c. RIP detection of the relation between miR-212-5p and SOD2; d. RT-qPCR and Western blot examination of SOD2. The data in the figure were all measurement data, and the manifestation of the values was mean ± SD (N = 3). * Vs. the Pro + mimic NC, *P* < 0.05.

RETRACTED

### 3.6 Augmented SOD2 partially turns around Pro’s impact on A2780 cells

To verify that Pro impacted the biological functions of A2780 cells via modulating circ-ZFR/miR-212-5p/SOD2 axis, PCDNA3.1-SOD2 and its NC (PCDNA3.1-NC) were transfected into A2780 cells treated with 20 μg/mL Pro. Verification of the transfection was implemented (Figure 6(a)). The experimental results elucidated the suppression of Pro on A2780 cell growth and glycolysis was partially turned around after augmenting SOD2 (Figure 6(b-g)). In short, Pro restrained A2780 cells’ biological functions via modulating circ-ZFR/miR-212-5p/SOD2 axis.

**Figure 6.** Augmented SOD2 partially turns around Pro’s impact on A2780 cells.

a. RT-qPCR and Western blot examination of SOD2; b. CCK-8 detection of cell proliferation; c. Flow cytometry examination of cell apoptosis; d. Western blot analysis of cleaved-PARP expression; e-f. Transwell test of cell migration and invasion; g. Glucose uptake, lactic acid, and ATP production. The data in the figure were all measurement data, and the manifestation of the values was mean ± SD (N = 3). * Vs. the Pro + PCDNA3.1-NC, *P* < 0.05.

## 4 Discussion

Numerous evidence has clarified Pro influences OC cell advancement via both direct and indirect means. For instance, Pro constrains OC cell proliferation and cisplatin resistance via mediating miR-374a/FOXO1 axis [15]. Pro suppresses MEK/ERK signal transduction via targeting the circVPS13C/miR-145 axis, thereby constraining OC cell advancement with movement [16]. In this research, Pro restrained OC cell progression with glycolysis dose-dependently in *vitro*. Additionally, the results of this study uncovered the novel regulatory mechanism of Pro on OC cell biological behavior, that is, Pro constrains OC cell progression via targeting the circ-ZFR/miR-212-5p/SOD2 axis.

As all known, glucose metabolism is a crucial source of energy, while metabolic plasticity enables cancer cells to reprogram to cope with cellular and environmental alteration, and is the extremely critical marker of malignant tumors [17]. Cancer cells are prone to make use of glucose at an exponential rate, namely AG, and tumor glycolysis is the crux to imperative management of cell biological energy and uninterrupted cancer growth [18]. As reported, the genomic instability of oncogenes and tumor suppressors are the hinges of this metabolic transformation [19]. This metabolic transformation has been testified in OC, which enables cancer cells to survive in an environment devoid of nutrients and oxygen, become tolerant to stress, and metastasize to different sites [20]. Several works have manifested Pro is available to influence AG in cancer. For instance, Pro destroys AG in lung cancer (LC) via modulating the circTADA2A/miR-455-3p/FOXM1 axis [21]. Pro disrupts AG in CRC cells via inactivating the NMDAR-CamKII-ERK pathway [22]. These studies illuminated Pro constrained cancer progression via disrupting AG. This study also testified to this viewpoint. The results elucidated Pro treatment repressed OC cell advancement in *vitro* and glucose uptake, lactic acid, and ATP production dose-dependently. These results manifested Pro constrained OC cells’ AG in *vitro*.

RETRACTED

Interestingly, Pro therapy distinctly reduced circ-ZFR in OC cells. Antecedent researches have illuminated circ-ZFR is augmented in diversified cancers like non-small cell LC [23], BC [14] and GC [24]. In the meantime, circ-ZFR was augmented in OC cells, and silenced circ-ZFR restrained OC cell advancement with glycolysis. Additionally, circ-ZFR was testified to modulate SOD2 via performing as a sponge for miR-212-5p. MiR-212-5p has been testified as a tumor suppressor in diversified cancers, covering triple negative breast cancer [25], clear cell renal cell carcinoma [26] and CRC [27]. Meanwhile, miR-212-5p was declined in OC cells, and elevated miR-212-5p repressed OC cell progression with glycolysis. This finding clarified miR-212-5p Might perform as OC’s tumor suppressor. Notably, this is not the first time that circRNA participates in OC’s physiological and pathological process via absorbing miRNA. For instance, circ_0002711 was augmented in OC tissues and cells, and repressive circ_0002711 restrained OC cell growth and AG via mediating miR-1244/ROCK1 axis [28]. CircRNA FGFR3 is augmented in OC patients and stimulates OC’s epithelial mesenchymal transformation via modulating miR-29a-3p/E2F1 axis [29].

Antioxidant SOD2, a conserved antioxidant enzyme, is available to remove mitochondria-produced reactive oxygen species and exerts a critical role in maintaining cell homeostasis [30]. Elevated SOD2 is associated with unpleasing prognosis, metastasis, and malignant progression of diversified cancers [31]. Several foregoing researches have illuminated SOD2 as augmented by epithelial ovarian cancer (EOC) tissues and cells, accelerating EOC cell advancement with chemical sensitivity [32]. Meanwhile, SOD2 was elevated in OC cells, and augmented SOD2 partially turned around Pro’s repression on OC cells, and boosted OC cell progression with glycolysis. These results elucidated Pro constrained OC cells’ biological functions via mediating circ-ZFR/miR-212-5p/SOD2 axis.

RETRACTED

Several limitations were presented in this research. For one, whether circ-ZFR and miR-212-5p were available to be adopted as OC latent biomarkers should be further detected in the blood of OC patients and their association with clinicopathology. Further, in *vivo* animal experiments should be further implemented to verify Pro’s action on OC tumor growth via modulating circ-ZFR/MiR-212-5p/SOD2 axis.

## 5 Conclusion

In brief, this study uncovers the latent mechanism by which Pro constraints OC cells’ AG via targeting the circ-ZFR/miR-212-5p/SOD2 axis, elaborating that Pro is provided with latent value in OC treatment.
